The article "A Novel Framework for Melanoma Lesion Segmentation Using Multiparallel Depthwise Separable and Dilated Convolutions with Swish Activations" was published in 2023. Journal: J Healthc Eng.

# A Novel Framework for Melanoma Lesion Segmentation Using Multiparallel Depthwise Separable and Dilated Convolutions with Swish Activations

**DOI:** 10.1155/2023/1847115

**Published:** 2023-02-06

**Authors:** Maryam Bukhari, Sadaf Yasmin, Adnan Habib, Xiaochun Cheng, Farhan Ullah, Jaeseok Yoo, Daewon Lee

**Affiliations:** ^1^Department of Computer Science, COMSATS University Islamabad, Attock Campus, Attock, Pakistan; ^2^Department of Computer Engineering, UET Taxila, Taxila, Pakistan; ^3^Department of Computer Science, Swansea University, Bay Campus, Fabian Way, Swansea SA1 8EN, Wales, UK; ^4^School of Software, Northwestern Polytechnical University, Xian 710072, China; ^5^Graduate School of Advanced Imaging Science, Chung-Ang University, Seoul, Republic of Korea; ^6^School of Art and Technology, College of Art and Technology, Chung-Ang University, Seoul, Republic of Korea

## Abstract

Skin cancer remains one of the deadliest kinds of cancer, with a survival rate of about 18–20%. Early diagnosis and segmentation of the most lethal kind of cancer, melanoma, is a challenging and critical task. To diagnose medicinal conditions of melanoma lesions, different researchers proposed automatic and traditional approaches to accurately segment the lesions. However, visual similarity among lesions and intraclass differences are very high, which leads to low-performance accuracy. Furthermore, traditional segmentation algorithms often require human inputs and cannot be utilized in automated systems. To address all of these issues, we provide an improved segmentation model based on depthwise separable convolutions that act on each spatial dimension of the image to segment the lesions. The fundamental idea behind these convolutions is to divide the feature learning steps into two simpler parts that are spatial learning of features and a step for channel combination. Besides this, we employ parallel multidilated filters to encode multiple parallel features and broaden the view of filters with dilations. Moreover, for performance evaluation, the proposed approach is evaluated on three different datasets including DermIS, DermQuest, and ISIC2016. The finding indicates that the suggested segmentation model has achieved the Dice score of 97% for DermIS and DermQuest and 94.7% for the ISBI2016 dataset, respectively.

## 1. Introduction

Melanoma is a severe kind of skin cancer with a very high mortality rate. Although there are only 2% of all the skin cancer types, melanoma is responsible for 75% of deaths occurred due to skin cancer [1]. In USA only, about 87,110 new cases are reported every year out of which 9,730 patients lose their lives due to this lethal skin cancer [2]. Similarly, in 2016 a total of 6,800 fatalities due to melanoma were reported in Canada [3]. Usually, the exposed regions of skin to sunlight are highly affected by melanoma e.g., face, legs, and arms. The borders and colors of melanoma moles are uneven and evolving which represent the severity level of the disease [4]. Many advanced techniques for the treatment of skin cancer are available including radiation therapy and immunotherapy. In clinical practice [5], these techniques are combined with surgery but still the survival rate of advanced stages of melanoma is quite low and is around 15%. On the other hand, the survival rate for the early stages of melanoma is around 95% [6]. In order to diagnose the medical problems of melanoma lesions, dermatologists directly examine the damaged skin's uniformity, inconsistencies in the borders, and color changes [4]. Moreover, dermoscopy, a nontrauma skin imaging technique, is also very popular to assist dermatologists to examine the affected skin. The accuracy for identification of melanoma lesions through dermoscopy is higher than the traditional method of ABCD rule criteria [7]. This ABCD rule is designed by the American Society for skin lesions [8]. Nevertheless, the biopsy test is the only thing on which the performance is solely dependent. In the initial stages, the identification of melanoma greatly matters since in the initial stages the possibility of recovery is much higher than in the later stages. However, the manual identification of melanoma needs an expert dermatologist followed by a stage in which the decision is made to assess a subjective variation.

Numerous researchers have proposed to automate the analysis process and extend the knowledge that can identify lesions accurately and helps different healthcare systems which are based on the Internet of Things (IoT) [9–11]. There exist traditional techniques, e.g., Otsu and Stochastic, that can perform melanoma segmentation, but these thresholding techniques are not the end-to-end solution, and owing to artifacts, this might lead to under or over segmentation problems. Therefore, there is a need for automated systems to automatically diagnose skin lesions for the treatment of skin cancer patients. The lighting conditions and different orientations also make it a challenging task for automated systems to analyze them [12]. Some researchers highlighted these issues recently and observed that there is very low diagnostic accuracy due to the presence of these issues in clinical images [13].

Recently, deep-learning approaches are also utilized for the task of automated skin lesion segmentation to overcome the challenges with traditional methods. The performance of these deep-learning-based methods is exceptional in segmenting skin lesions as compared to the traditional dermatologists [1]. A lot of deep-learning-based segmentations are proposed in the existing research studies for skin lesions, but there is still space to enhance the algorithms in terms of both parameters and performance [14–17].

From this line of research, we proposed an efficient deep-learning model for end-to-end segmentation of melanoma lesions to overcome all the challenges which include intraclass variations and lighting conditions as well as other related issues. The proposed framework uses the UNet architecture as the base architecture for end-to-end segmentation of melanoma lesions, as it has a very strong capability in biomedical image segmentation [18]. More explicitly, it consists of a downsampling path, a bottleneck layer, and an upsampling path. The downsampling path consists of multidilated convolution blocks (MDC) and depthwise separable convolutions blocks (DSC) that empower the process of feature learning across the channels on the image. The parameters of convolution are dramatically reduced with these depthwise separable convolutions without compromising the performance. The generalization ability of the model is improved by these convolutions while avoiding overfitting. Spatial and cross-channel correlations are also separated with the help of these convolutions. Moreover, there is the use of swish activations in the MDC block. The nonmonoatomic property of swish is very advantageous in deep-learning algorithms. All these characteristics make the proposed framework more reliable in segmenting melanoma lesions. The following points describe our contribution:

- The proposed approach is capable of localizing melanoma lesions and multiple types of cancer in a single image by designing DSC blocks with multidilated features
- The proposed segmentation model accurately segments the lesions by overcoming the challenges presented in the ISBI2016 dataset
- We used skin refinement as a preprocessing step to eliminate artifacts from dermoscopic images.

The rest of the paper is organized in the following way: Section 2 thoroughly explains the review of current approaches.  Section 3 explains our proposed methodology in detail.  Section 4 explains the experimental details, results, and discussion. Lastly, Section 5 provides the conclusion of the paper.

## 2. Literature Review

The segmentation of melanoma lesions is a fundamental technique in designing the automated detection model of skin cancers. Since the segmentation of lesions plays an important role in the classification task of skin cancer [19–21]. Automated segmentation techniques are further split into traditional and deep-learning techniques, along with some advanced hybrid deep learning models. The following is a critical literature assessment of each kind of method in the segmentation of melanoma lesions.

The conventional techniques of melanoma lesions segmentation mostly involve iterative selection [22, 23], adaptive threshold [24], iteration merging of regions [25], and Otsu threshold [26]. Nevertheless, as a result of the existence of artifacts in dermoscopic images the effectiveness of thresholding-based techniques will be diminished [22, 26]. In [26], the accuracy of the proposed algorithm is acceptable but the images that were segmented have uneven borders as well as reduces the resolution of the images. In [27], the authors suggested a method to address the challenges that arise in [26]. Another collection of studies [25, 28] suggested a region merging technique to perform segmentation. In this method, the identical regions of the images are clustered together. To overcome the challenges of color, low contrast, and illustration, the region merging technique performs well. In [25], lesion segmentation is carried out by these identical regions having identical attributes. Overall, these approaches need a lot of manual parameter tuning, such as threshold values in thresholding-based segmentation, making them unsuitable for automated CAD systems.

Another research group [29–32] suggested deep-learning techniques for segmentation and achieved considerable outcomes as compared to the standard methods. In [31], an FCRN, i.e., fully convolutional-residual-network was suggested to address the challenges of model overfitting in the task of melanoma segmentation. In [32], localization of lesions is accomplished by utilizing the region-based CNN followed by the machine learning fuzzy-clustering technique. In [29], a 19-layer CNN is designed to improve and enhance the results of melanoma segmentation. More specifically, in this study, Jaccard distance is utilized as a loss function. With the assistance of this loss function, the segmentation performance improves and also the problem of overfitting arises between normal and melanoma images. In [30], FRCN, i.e., full CNN was designed for segmentation of melanoma lesions. In order to segment, the lesion areas of different scales a segmentation model based on multiscale convolution is proposed in [33] which efficiently extracts the areas of lesions. A multistage segmentation model was proposed in [34] to perform the end-to-end segmentation of skin lesions. They also combined and integrates the context information with their model. The boundary of lesion segmentation is further improved in [35]. They combined the mixed feature inputs and proposed a multibranch fusion network and performed an immense set of experiments to evaluate their model. In [36], a new method for automatic segmentation of skin lesions is designed which was capable of learning more powerful and distinguishable features. This model used cross-net-based aggregation. In [37], to segment lesions and lessen the impact of artifacts, a hybrid technique was suggested by integrating the convolutional and recurrent neural networks. Nevertheless, a two-stage object detection model such as RCNN produces about 2 thousand patches per image for lesion identification. Due to this reason, melanoma localization becomes computationally expensive in these approaches. Furthermore, while all of these deep-learning algorithms for lesion segmentation produce outstanding results, there is still a gap for improvement in terms of model performance.

In addition, to acquire more information features from dermoscopy images, some hybrid models are also designed such as in [38] for bilinear merging, they used ResNet and VGG to extract high-level features and trained their algorithm using SVM classifiers. They achieved the best accuracy results on several test sets. In order to cope with the intraclass inconsistency of lesions, a multiconvolution neural network is proposed in [39]. This model was combined with an adaptive sample strategy of learning. This technique also deals with related noise interference. In [40], encoded output features are converted into Fisher Vectors by using the weights of the pretrained model which is a deep residual network. They also used trained SVM to achieve the recognition task and have achieved a significant performance on a test set of classification challenges of ISBI2016. However, their approach was not an end-to-end solution and the overall architecture of the model was very complex. The advantages of hybrid approaches include improved performance and broader feature acquisition; nevertheless, the computational complexity of hybrid deep-learning models is high, making them slow.

## 3. Methodology

The detail of our proposed framework is presented in Figure 1. In this research, we have utilized three different datasets. The instances in the dataset undergo some preprocessing stages for improved quality images to remove artifacts like hair, bubbles, and other patches. This is followed by steps to localize the melanoma lesions.

### 3.1. Preprocessing

Before giving the input images to the deep-learning model, all the images are preprocessed to remove noises from them. This step is necessary for very precise segmentation. Most commonly used image preprocessing techniques involve image smoothing, resizing, identification of ROIs, and denoising of images. For the elimination of artifacts from dermoscopic images, Gaussian smoothing is the most effective technique. In the suggested method, we have performed the dilation followed by erosion also referred to as morphological closing. Later on, in the next stage, we performed the sharpening operations over the images to further enhance the quality of the images. Some sample images before and after preprocessing are depicted in Figure 2.

### 3.2. Data Augmentation

Usually, the publicly accessible training images for all categories are not dispersed evenly, resulting in the class imbalance issue [41]. In the suggested method, we increase the total number of samples in the train set by employing different types of augmentation such as flipping, cropping, and rotating.  Table 1 lists the different types of augmentation and their values used to augment the samples. More specifically, 15 additional images are sampled from a particular dermoscopic image by using the augmentation types given in Table 1. The main rationale to use this phase in our strategy is to reduce overfitting problems and improve the model's predictive performance.

### 3.3. Proposed Architecture

Our proposed framework consists of three major parts which include the downsampling path to down sample an image by extracting the features which represent what is present in an image followed by the bottleneck and upsampling path to upsample an image to get the localization of the required lesion in an image as shown in Figure 3(a). The complete architecture of each part is described below:

#### 3.3.1. Downsampling Path

The downsampling path of the model consists of a multidilated convolution (MDC) block and depthwise separable [30] convolution block (DSC) to encode features of melanoma lesions followed by max-pool operations of size 2 × 2 to reduce the spatial dimensions of the images as shown in Figure 3(a). The architecture of the MDC and DSC block are given in Figure 3(b). The feature extraction part starts from the regular convolution of size 1 × 1 and 3 × 3 max-pool on an input image of size 256 × 256 × 3 followed by ReLu [33] activation functions. Besides this, input is also given to the DSC block as shown in Figure 3(b). In the DSC block, the depthwise separable convolution of sizes 1 × 1 and 3 × 3 is performed on every channel of an input image independently. Afterwards, a 1 × 1 window is utilized as pointwise convolution to project to a new channel space after a channel is computed by depthwise convolution as shown in Figure 4. The depthwise separable convolutions are not like spatial separable convolutions which are also referred as “separable convolutions” in the community of image processing [42]. The mathematical formulation is given below:

(1) $$\begin{array}{c} Conv={\left(W,y\right)}_{\left(i,j\right)}=\overset{K,L,M}{\underset{k,l,m}{\sum }}W_{\left(k,l,m\right)}∙y_{\left(i+k,j+l,m\right)}\text{,}\\ PointWiseConv={\left(W,y\right)}_{\left(i,j\right)}=\overset{M}{\underset{m}{\sum }}W_{m}∙y_{\left(i,j,m\right)}\text{,}\\ DepthWiseConv={\left(W,y\right)}_{\left(i,j\right)}=\overset{K,L}{\underset{k,l}{\sum }}W_{\left(k,l\right)}⊙y_{\left(i+k,j+l\right)}\text{,}\\ SeparbleConv={\left(W_{p},W_{d,y}\right)}_{\left(i,j\right)}={PointWiseConv}_{\left(i,j\right)}\left(W_{p},{DepthWiseConv}_{\left(i,j\right)}\left(W_{d,y}\right)\right)\text{.} \end{array}$$

In the above equations, ⊙ shows the elementwise product. The benefit of depthwise separable convolutions over traditional convolutions is the total number of parameters [43]. For this, consider a standard convolution with a feature map **F** and suppose that value of stride and padding is one. This can be computed as the following equation:

(2) $$\begin{array}{c} F_{k,l,m}=\underset{i,j,m}{\sum }K_{i,j,m,n}∙I_{k+i-1,l+j-1,m}\text{.} \end{array}$$

For these standard convolutions, the total number of parameters and computational cost can be calculated as follows:

(3) $$\begin{array}{c} k\times k\times M\times N\;and\;k\times k\times M\times N\times H\times W\text{,} \end{array}$$

where the input image or input feature maps are represented by **I**, while **k** denotes the kernel of convolution with size **k** × **k**. The **M** and **N** denote the number of input and output channels while the height and width of input feature maps or input images are denoted by **H** and **W**, respectively. Furthermore, for depthwise separable convolutions which is a combination of depthwise and pointwise convolutions, the output feature maps are calculated as follows:

(4) $$\begin{array}{c} F_{k,l,n}^{,}=\underset{i,j}{\sum }K_{i,j,m}^{,}∙I_{k+i-1,l+j-1,m}\text{.} \end{array}$$

Similarly, for these depthwise separable convolutions, the total number of parameters and computational cost is calculated as follows:

(5) $$\begin{array}{c} k\times k\times M+M\times N\;and\;k\times k\times M\times H\times W+M\times N\times H\times W\text{.} \end{array}$$

Now, in order to compare the parameters of both types of convolutions, we obtained the following equation:

(6) $$\begin{array}{c} \frac{k\times k\times M+M\times N}{k\times k\times M\times N}=\frac{1}{N}+\frac{1}{k^{2}}\text{.} \end{array}$$

It can be shown and seen that the number of parameters is about 8 to 9 times less in depthwise separable convolutions than in standard convolutions. Hence, it is observed that we improved the network without an extensive increase in the number of parameters of the network and also empowered the network to learn deep dilated features which in turn gives more contextual information. Moreover, the output of regular convolutions and max-pool are concatenated and given as input to the first dilated convolution in the MDC block as shown in Figure 3(b). Similarly, the input of second and third dilated convolutions in the MDC block is the output of regular convolutions, max-pool, and the result of previously dilated convolution. Furthermore, in the MDC block, three convolution operations utilizing the dilated filters of size 1 × 1, 2 × 2, and 3 × 3, respectively, are used. The convolutions which use the dilated filters are also called dilated or atrous convolutions. For these, a dilated filter **w** also called kernel is convolved over the input signal, and for each location, **i** is the output, and **y** is computed by equation (7), ([44])

(7) $$\begin{array}{c} y\left[i\right]=\underset{k}{\sum }x\left[i+r∙k\right]w\left[k\right]\text{.} \end{array}$$

In equation (7) the *r* is representing the value of the stride by which the input signal is sampled which is a similar operation to convolve over any input signal *x* with the help of filters *w* that are upsampled by inserting *r* − 1 zero along each spatial dimension that are consecutive. These are very helpful as a large receptive field of view is enhanced by dilated convolutions of the given input image. After each dilated convolution in the MDC block, there is the use of batch normalization [31] and swish activations [32] as shown in Figure 3(b). The use of batch normalization [31] fastens the training process and prevents the model from overfitting. A dropout layer of rate 0.05 is also added after every max-pool operation. Furthermore, the swish activations are defined as [45]

(8) $$\begin{array}{c} f\left(x\right)=x∙\sigma \left(x\right)\text{.} \end{array}$$

In equation (8), the *σ*(**x**)=(1+exp (−**x**))^−1^ represents the sigmoid function. This activation function is bounded below and unbounded above. The properties of swish activation include that it is smooth and the property of non-monotonicity which distinguishes it from other activation functions. The derivative of the swish is given below in equation (9) [45]

(9) $$\begin{array}{c} {f\left(x\right)}^{,}=\sigma \left(x\right)+x∙\sigma \left(x\right)\left(1-\sigma \left(x\right)\right.\\ =\sigma \left(x\right)+x∙\sigma \left(x\right)-x∙\sigma {\left(x\right)}^{2}\\ =x∙\sigma \left(x\right)+\sigma \left(x\right)\left(1-x∙\sigma \left(x\right)\right)\\ =f\left(x\right)+\sigma \left(x\right)\left(1-f\left(x\right)\right.\text{.} \end{array}$$

Moreover, the output of MDC blocks is concatenated to depthwise convolution blocks, and the result of regular convolutions and max-pool is shown in Figure 3(b). The number of filters set for each of our convolution blocks is 16, 32, 64, and 128, respectively. Moreover, the starting weights for regular convolution and convolutions in MDC blocks are initialized with “He normal” weight initialization which is defined as [46, 47]

(10) $$\begin{array}{c} W∼\;G\left(0,\sqrt{\frac{2}{n}}\right.\\ Or\;W\left[i\right]=RandomUniform\left(low\right.=-limit,high=limit,size=\left(F_{in},F_{out}\right)\text{.} \end{array}$$

In the above equation (10), **G** is just a random number with Gaussian probability distribution while the total number of inputs coming towards a particular neuron is represented by **n**. Furthermore, $\sqrt{2/n}$ is used to calculate the standard deviation while the 0 represents the mean. In addition, **F**_**in**_ and **F**_**out**_ are the number of inputs and outputs to the layer, respectively. Similarly, the weights of depthwise separable convolutions are initialized with the Glorot weight initialization method which is also called Xavier initialization. The main objective of the downsampling path is to extract features that describe the semantics of the image with loss of spatial and localization information.

#### 3.3.2. Bottleneck Path

The bottleneck path of the proposed framework consists of 1 × 1 and 3 × 3 convolution followed by depthwise separable convolution block (DSC) and MDA blocks as shown in Figure 3(a). The resulting feature maps of the last max-pool operation on an input image in the downsampling path are given as inputs to the bottleneck path which yields output feature maps of dimension 16 × 16 × 2323. These resulting feature maps are then given as input to the very the first layer of the upsampling path to localize the melanoma lesion.

#### 3.3.3. Upsampling Path

The upsampling path of the model consists of transposed convolution with kernel sizes of 3 × 3 with a stride of 2 × 2 followed by the operation of concatenation to corresponding convolution blocks of downsampling path as shown in Figure 3(a) to combine the context and localization information to segment out the melanoma lesions. Transposed convolutions are the reverse processes of convolution, and it is more robust than simple upsampling as it fills up the details with proper learning. These are also called fractionally stride convolutions. Moreover, the concatenation operations between upsampling and downsampling path at the appropriate position help to restore the localization information that is lost during downsampling an image. So more specifically, the input from the bottleneck layer is first given as an input to the first transposed convolution layer. Then, by means of skip connections, the output generated from this layer is concatenated to the last MDC and DSC blocks downsampling path. Moreover, this process is repeated three more times. In the end, the output of the last MDC and DSC blocks in upsampling path is passed through 1 × 1 convolution followed by sigmoid activation to get the required segmented image of the lesion.

## 4. Experiments, Results, and Discussion

In this section, we discuss the datasets used for experimentation purposes and evaluation metrics used to evaluate the model as well as results of the model. In addition, the proposed model is designed in the Keras framework available in Python, and simulations are run on Google Colab with 12 GB RAM and NVIDIA Tesla K80 GPU. The hyperparameters of the model include the weight initialization, weight optimizer, learning rate, and epochs which are set to Xavier, Adam, 0.001, and 150, respectively.

### 4.1. Datasets

To assess the universality of our proposed model, we evaluated it on three distinct datasets, i.e., DermIS, DermQuest, and ISBI2016. All the datasets contain skin lesion images in RGB format. More explicitly, the DermQuest contains 152 melanoma images while 122 images belong to the nevus class. Similarly, in DermIS, the total number of melanoma class images is 43 while the nevus class has a total of 26 images. The DermQuest and DermIS datasets contain a limited number of images, so augmentation is applied to the training set. Moreover, the dataset ISBI2016 comprised 900 melanoma images in the train set and 379 images in the test set. The train and test division of images are already provided by the dataset publisher. For a fair comparison, we utilize the same train and test sets.

### 4.2. Performance Evaluation Metrics

To examine the performance of the model, we utilized different evaluation metrics [48–51] including dice score, specificity, sensitivity, and Jaccard score. The following equations (11)–(15) are used to compute these metrics

(11) $$\begin{array}{c} Accuracy=\frac{TP+TN}{TP+TN+FP+FN}\text{,} \end{array}$$

(12) $$\begin{array}{c} Dice\;score=\frac{2\times TP}{2\times TP+FP+FN}\text{,} \end{array}$$

(13) $$\begin{array}{c} Specificity=\frac{TP}{TP+FP}\text{,} \end{array}$$

(14) $$\begin{array}{c} Sensitivity=\frac{TP}{TP+FN}\text{,} \end{array}$$

(15) $$\begin{array}{c} Jaccard\;score=\frac{TP}{TP+FP+FN}\text{,} \end{array}$$

where TP denotes the true positives, FP denotes the false positives, TN denotes the true negatives, and FN denotes the false negatives.

### 4.3. Results of DermIS Dataset

In the first step, we evaluate the proposed model on the DermIS datasets containing melanoma and nevus class images along with their mask images. As previously stated, artifacts like hair, air bubbles, and other noises can be seen in the images of the DermIS dataset. The existence of these types of artifacts will influence performance accuracy. To address this problem, we have performed the preprocessing on images that are discussed in Section 3.1. In addition, we have also performed the data augmentation described in Section 3.2 to increase the number of training samples since DermIS has a very limited number of images. This is done to expand the number of instances since a minimal amount of training data leads to overfitting issues. In Figure 5, the results of augmentation are depicted. The proposed model takes the dermoscopic images along with their ground truth images as input and outputs the segmented images. The results of melanoma segmentation are depicted in Figure 6 along with their actual ground truth images and contour images.

Column (A) in Figure 6 shows the original images that were preprocessed. Column (B) shows the actual ground truth images. Following on, column (C) shows the contour images of actual ground truth images. The contour is shown by the red borders in column (C). Column (D) depicts the output of the segmentation model in form of segmented images while column (E) shows the output images with contours. The effectiveness of the proposed method on this database was assessed utilizing previously defined metrics. As shown in Table 2, the Dice score achieved for this dataset is 97% which shows the robustness of our model performance in localizing skin lesions. The accuracy and Jaccard indexes are 97% and 94% while sensitivity and specificity are 93%.

### 4.4. Result of DermQuest Dataset

In the second step, we evaluated the performance of the proposed model on the DermQuest dataset. All of the trials on this data, like the DermIS dataset, make use of melanoma images and associated ground truth images. More specifically, we first perform the preprocessing step over the images to eliminate the noises in the form of artifacts. The number of images in this dataset is also less in number; hence, we also perform the data augmentation on this dataset. The results of melanoma segmentation for the DermQuest dataset are depicted in Figure 7 along with their actual ground truth images and contour images. Column (A) in Figure 6 shows the original images, column (B) shows the actual ground truth image, and column (C) shows the contour images of actual ground truth images. Moreover, column (D) depicts the output of the segmentation model in form of segmented images while column (E) shows the output images with contours. For this dataset, we have achieved the highest Dice score, accuracy, and Jaccard score in comparison with the DermIS dataset. The proposed model achieved the Dice score of 97% and the Jaccard score of 96% in localizing the melanoma lesions. Moreover, the accuracy, sensitivity, and specificity attained for this dataset are 98%, 90%, and 95%, respectively.

### 4.5. Results of ISBI2016 Dataset

The suggested framework's efficacy was also examined using benchmark datasets namely ISBI 2016 by “International Symposium on biomedical images (ISBI) in the challenge of skin lesion analysis towards melanoma detection” [52]. For the challenge of segmentation, this database comprises a total of 1,279 images out of which 900 images belong to the train set while the remaining 379 images belong to the test set. All dermoscopic images in this dataset, like those in DermIS and DermQuest, go through the preprocessing stage. The total number of training images in this dataset is sufficient for training purposes; hence, there is no data augmentation is applied to this dataset.  Figure 8 shows the segmentation results of the proposed algorithm on the ISBI2016 dataset. In Figure 8, column (A) shows the original test images with their ground masks shown in column (B). The test images with contour around the boundary are shown in column (C). The predicted mask and output with contour are shown in columns (D) and (E) of Figure 8, respectively. In the test set of this dataset, there are more challenging images. As shown in row 1 of Figure 8, the lesion area of the first image has very similar to normal skin but still, it can be accurately segmented by a model as shown in row 1 column (D) of Figure 8. The boundaries of lesions are still more distilled and smooth. The evaluation scores achieved by our proposed model on this dataset include a Dice score which is 94.7%, a Jaccard score of 90%, and an accuracy of 95%, respectively. Moreover, the sensitivity and specificity achieved for this dataset are 92% and 90%, respectively.

We also compared our results with challenge winners of ISBI2016. In this challenge, almost 28 groups provide their results, as listed in Table 2. This ISBI ranked the competition participants based on their best average Jaccard score. Due to the precise segmentation of deep-learning models, it is observed from Table 2 that most of the participants in the competition employ deep-learning techniques. For instance, AlexNet, VGG16, and ResNet-based pretrained models are utilized to approximate the edges and boundaries of lesions.

It is evident from Table 2 that the proposed algorithm attained the highest results among challenge winners. The comparison with all challenge winners and the proposed framework is given in Table 2 and is graphically presented in Figure 9. In terms of the Jaccard score, the proposed model has a very remarkable performance over the top two participants. The Dice score of the proposed model is also improved among all challenge winners. Moreover, the scores of each test set image in the ISBI2016 dataset are shown in Figure 10. It is observed from Figure 9, that most of the test samples achieved greater than 80% Dice, Jaccard, and accuracy scores. There are only a few samples in which the Jaccard score falls below 50%. Moreover, to consider the effect of class unbalancing, we calculate the Dice and Jaccard score in three different ways. First, we consider no averaging method and calculate the scores; in the second way we consider the average method of “micro” (mi) which globally calculates the FP, FN, and TP without favoring any class. Similarly, in the third way, we use the average method of “macro” (ma) in which we calculate the scores separately for both background and foreground classes. It is observed from the results that our proposed framework significantly addresses the challenges of segmentation in skin lesions which includes intraclass differences and visual similarity of lesion features with normal skin.

Furthermore, the training graphs of accuracy and loss of the model for all three datasets are also shown in Figure 11. In general, the accuracy of the model is used to determine the total number of correct predictions. The higher value of accuracy shows the better capability and performance of the model. The graphical representation of accuracy is shown in Figure 11, and it is observed that during training the model achieves an accuracy greater than 90%. Similarly, model loss values during training of all three datasets are also plotted. The predictions of the model are more accurate if the loss of the model is near to zero. It is observed that the loss values of the proposed model on all three datasets are near zero. The x-axis of Figure 11 shows the total number of epochs while the y-axis shows the accuracy and loss values epoch by epoch of the proposed model. Moreover, during the training of the deep-learning model, when an input image passes through successive layers of architecture; then, each layer gives output in the form of feature maps of different dimensions. These feature maps indicate how your model encodes and learns the features of images layer by layer. Usually, in the starting layers, the model extracts low-level features while subsequently more high-level features are extracted. The activation maps of some intermediate layers of the proposed algorithm are also shown in Figure 12.

Figure 12 illustrates that lesion areas are more focused on the proposed model. This indicates that the model learns more effective and discriminative features of lesion areas in the given image.

### 4.6. Comparative Analysis with State-of-the-Art Approaches

We have compared the performance accuracy of our proposed framework with other state-of-the-art approaches. It is noticeable from Table 3 that recent approaches use many deep-learning approaches to automatically segment melanoma lesions. Bozorgtabar et al. [53] proposed an unsupervised method for skin lesion segmentation. In this work, the information about the context of the image is exploited at the superpixel level. They achieved Dice and Jaccard scores of 0.86% and 0.66%, respectively. Similarly, Yaun et al. [29] proposed a19-layer deep convolutional network for automatic segmentation of skin lesions. In their work, the proposed model is trained with a loss function of Jaccard distance and achieved Dice and Jaccard scores of 91% and 84%, respectively, which is very much better. Furthermore, Li et al. [43] proposed a dense convolutional neural network based on residual learning for skin lesion segmentation. They achieved a Dice score of 93% with an 87% Jaccard score. Rashid et al. [40] proposed a two-stage method and utilized the approach of object detection algorithms named single shot detector (SSD) for localization of melanoma lesion followed by a second stage in which level set algorithm is used to segment the melanoma lesion. The Jaccard and Dice scores achieved by their approach are 90% and 82%, respectively. Moreover, Tang et al. [34] proposed a new novel multistage UNet-based model combined with context information fusion structure (CIFS) for melanoma segmentation and achieved an appropriate improvement in the Jaccard score. In comparison with all the previous approaches, our model outperforms especially in terms of Jaccard analysis. Wei et al. [45] proposed an ensemble lightweight neural network for melanoma segmentation and achieved a significant and excellent performance in Dice and Jaccard scores which are 96% and 92%, respectively. The main reason for having efficient performance results is the end-to-end automatic segmentation of melanoma lesions by employing the use of (DSC) blocks with multidilated filters which enlarges the receptive field and view of filters. Moreover, the nonmonoatomic property of swish activation makes the training smooth. Furthermore, in our approach, we applied a preprocessing technique on images that removes the artifacts in data that hinder the accurate segmentation of melanoma.

Table 3 represents the comparison between the existing techniques and the proposed framework. From Table 3, it is observed that there is significant improvement found in terms of Jaccard and Dice scores, especially in ISBI2016, which contains 379 challenging test images.

### 4.7. Discussion

Melanoma lesion segmentation remains one of the most difficult tasks in dermoscopy image analysis. Traditional segmentation methods such as Ostu and thresholding perform well but fails when artifacts and noises are observed in the images. In addition, they also require manual tuning of parameters such as threshold values. These manual settings limit their use in automated CAD systems. More explicitly, in CAD systems end-to-end solutions are preferable. Hence, in this research study, we proposed a deep-learning-based segmentation model to automatically segment the lesion from given dermoscopic images. The proposed model first encodes the dermoscopic images to extract the features of melanoma lesions using a DSC block in which depthwise separable convolutions are applied channelwise and has a smaller number of weights in comparison with the conventional convolutions. Following the activation function, swish is applied to achieve the nonlinearity on the resulting feature maps. In subsequent steps, the bottleneck layers are inserted followed by an upsampling path called a decoder to generate the segmented image containing the lesions. The proposed model performs well since it avoids the problems of overfitting by using convolution layers with fewer parameters using DSC blocks as well as by disentangling spatial and cross-channel correlations. The results presented in Table 2 provide accuracy, Dice score, Jaccard score, sensitivity, and specificity of the proposed model in comparison with challenge winners of the ISBI2016 dataset. Similarly, Table 3 provides a comparison with different research studies. The proposed method's strength is that it accurately segments out lesions from dermoscopic images of not only melanomic type cancer but also nevus type cancer whose images are available in DermQuest and DermIS datasets. This indicates the generalizability of the proposed method in terms of segmenting different types of lesions. In addition, the proposed method is less complex in comparison with the hybrid models that are large in terms of parameters. This is due to the adoption of DCS blocks in which depthwise separable convolutions are used to extract features with fewer number weights. However, one potential limitation of the method is that the model training is done from scratch, which takes long time for optimal convergence; thus, what if the encoder is set to pretrained weights? This would be an excellent future direction for this work. Furthermore, more challenging ISBI datasets on skin cancer should be utilized to investigate the performance.

## 5. Conclusion

Melanoma lesion segmentation is a very challenging task in the medical imaging domain since the normal and affected regions have the same appearance, and usually, the presence of artifacts and other noises in data decreases the segmentation performance. To address this challenge, different traditional segmentation methods are suggested by various researchers; however, these methods are not suitable for automated CAD systems due to many manual parametric steps. Therefore, we proposed a deep-learning-based segmentation model for automated segmentation of melanoma lesions from dermoscopic images. The suggested model employs the depthwise separable convolution blocks (DSC) which can learn the features from each space of an image. Moreover, multidilated filters broaden the view of kernels or filters and capture the information with large receptive fields. The use of swish activation proved to be very beneficial due to its nonmonoatomic behavior. The experimentation has been done on three different datasets including DermIS, DermQuest, and ISBI2016 datasets. The Dice and Jaccard scores for DermIS are 97% and 94%, for DermQuest are 97% and 96%, and for ISIC2016 are 94.7% and 90%, respectively. Future work will entail in improving the segmenting model by adding the attention modules such as CBAM and expanding the number of samples in training data in terms of challenging images.

## Figures and Tables

**Figure 1:** A schematic overview of the proposed methodology.

**Figure 2:** Image enhancement on ISBI2016 dataset; row 1 depicts the original dataset images, row 2 depicts the images after closing morphological operation, and row 3 depicts results after sharpening.

**Figure 3:** Architecture of proposed segmentation model.

**Figure 4:** Depthwise separable convolutions.

**Figure 5:** Results of augmentation on DermQuest dataset.

**Figure 6:** Results of melanoma segmentation on DermIS dataset.

**Figure 7:** Results of melanoma segmentation DermQuest dataset.

**Figure 8:** Sample melanoma segmentation results of ISIC2016 dataset from the skin with the respective masks and contour images.

**Figure 9:** Comparison in terms of accuracy, Jaccard, and Dice scores with challenge winners.

**Figure 10:** Segmentation performance of each test image in the ISBI2016 dataset.

**Figure 11:** Loss and accuracy graphs of each dataset during training.

**Figure 12:** Results of channel activation of intermediate layers of the model.

**Table 1:** Data augmentation types and their parameters.

Sl. no.	Augmentation types	Parameters
1	Rotate	90°, 180°, 270°
2	Crop from right	45°, 60°, 90°
3	Crop from left	45°, 60°, 90°
4	Crop from top	45°, 60°, 90°
5	Crop from bottom	45°, 60°, 90°
6	Flipping	Left right
7	Shifting	Shifted by (25, 25) pixels

**Table 2:** Results of skin lesion segmentation in ISBI2016 challenge.

Technique	Accuracy	Dice score	Jaccard score	Sensitivity	Specificity
ExB	0.95	0.91	0.84	0.91	0.965
CUMED	0.94	0.897	0.829	0.911	0.957
Mahmudur	0.952	0.895	0.822	0.88	0.969
SFU-mial	0.944	0.885	0.811	0.915	0.955
TMU team	0.946	0.888	0.81	0.832	0.987
UiT seg	0.939	0.881	0.806	0.863	0.974
IHPC-CS	0.938	0.879	0.799	0.91	0.941
UNIST	0.94	0.867	0.797	0.876	0.954
JoseLuis	0.934	0.869	0.791	0.87	0.978
Marco Romelli	0.936	0.864	0.786	0.883	0.962

Proposed	0.95%	0.90% (None)	0.82% (None)	0.92%	0.90%
	0.95%	0.947% (mi)	0.90% (mi)	0.92%	0.90%
	0.95%	0.92% (ma)	0.86% (ma)	0.92%	0.90%

**Table 3:** Comparison with state-of-the-art approaches.

Techniques	Accuracy	Dice score	Jaccard score	Specificity	Sensitivity
Rashid et al. [40]	0.90	0.901	0.82	0.98	0.83
Yaun et al. [29]	0.955	0.912	0.847	0.966	0.918
Li et al. [43]	0.959	0.931	0.870	0.96	0.95
Wei et al. [44]	0.962	0.923	0.867	0.974	0.934
Tang et al. [34]	0.95	0.91	0.85	0.96	0.92
Bozorgtabar et al. [53]	—	0.86	0.67	—	—
DermQuest	0.98	0.97	0.96	0.95	0.90
DermIS	0.972	0.97	0.94	0.93	0.93
ISBI2016	0.95	0.947	0.90	0.90	0.92

## Data Availability

The data used to support the findings of this study are publicly available.
